# Clinical significance of long noncoding RNA SPRY4‐IT1 in melanoma patients

**DOI:** 10.1002/2211-5463.12030

**Published:** 2016-02-03

**Authors:** Teng Liu, Song‐Ke Shen, Jian‐Gui Xiong, Yuan Xu, Han‐Qi Zhang, Hai‐Jun Liu, Zheng‐Gen Lu

**Affiliations:** ^1^ Department of DermatologyThe People's Hospital of ChizhouChina; ^2^ Department of DermatologyThe First Affiliated HospitalAnhui Medical UniversityHefeiChina; ^3^ Department of DermatologyWanbei Coal‐Electricity Group General HospitalSuzhouChina; ^4^ Department of InfectionNo. 2 People's Hospital of FuyangChina

**Keywords:** long noncoding RNA, melanoma, overall survival, SPRY4‐IT1

## Abstract

Long noncoding RNA SPRY4‐IT1 has been reported to promote melanoma cell growth and invasion, and to block apoptosis. The purpose of this study was to investigate the clinical significance of SPRY4‐IT1 in patients with malignant melanoma. The relative expression levels of SPRY4‐IT1 were measured in plasma samples from 70 patients and 79 healthy controls by quantitative reverse transcriptase polymerase chain reaction. SPRY4‐IT1 expression is high in melanoma patients but low in healthy controls, and is closely associated with tumor site and tumor stage. Elevated SPRY4‐IT1 significantly reduces overall survival rates of patients and is considered as an independent prognostic factor in patients with melanoma. The prognostic nomogram shows a good prediction of the probability of 5‐year overall survival of patients with melanoma (c‐index: 0.72). The calibration curve for the probability of survival presents good agreement between actual outcomes and predictive consequences. In summary, SPRY4‐IT1 may be a potential prognostic marker and a potential therapeutic target.

**Abbreviations**
AUC: area under curve
c‐index: concordance index
HOTAIR: HOX antisense intergenic RNA
lncRNA: long noncoding RNA
MALAT1: metastasis‐associated lung adenocarcinoma transcript 1
MEG3: maternally expressed 3
miRNA: microRNA
OS: overall survival
SPRY4‐IT1: Sprouty4‐Intron 1

Melanoma is a malignant tumor of melanocytes and a major cause of all skin cancer deaths 1. The clinical outcomes of melanoma are good when it is detected early. Accurate diagnostic tests for its early detection would therefore be useful. Despite substantial progression in the early detection and treatment of malignant melanoma, the overall survival (OS) remains poor, especially in patients with AJCC stage IV disease 2 due to its rapid progression and metastasis after surgery. It is essential to seek an effective biomarker to detect it at an early stage. To further understand the underlying mechanisms contributes to find a useful marker to diagnosis early and predict prognosis.

Mounting evidence showed that multiple complex changes are involved in the carcinogenesis and progression of melanoma, such as signaling pathways that control cell proliferation and apoptosis 3, genetic predisposition 4, and epigenetic regulation 5. A series of protein‐coding genes have been determined as potential diagnostic and prognostic biomarkers 6, 7.

Meanwhile, noncoding RNAs, lack of protein‐coding capacity, are commonly classified as small or long based on a nucleotide length. Small ncRNAs (microRNA, miRNA) are broadly conserved and involved in the transcriptional and post‐transcriptional regulation of genes through specific binding to 3′ untranslated region of their target mRNAs or transcripts 8, 9. In contrary to miRNA, long noncoding RNAs (lncRNA) are less well conserved and control gene expression by multiple mechanisms, especially epigenetic mechanisms 10. Emerging data supported that long noncoding RNAs (lncRNAs), more than 200 nucleotides in length, play a critical role in human disease and development 11, 12, 13. LncRNAs directly regulate chromatin regulatory proteins and modulate the activity of their interacting partners to impact target gene expression 14, 15. LncRNAs expression is dysregulated in various diseases, including heart disease 16, Alzheimer's disease 17, and psoriasis 18. The dysregulation of lncRNAs has been identified in various cancers, such as breast cancer 19, colorectal cancer 20, prostate cancer 21, and leukemia 21. Furthermore, lncRNAs have oncogenic or antioncogenic functions to control carcinogenesis and progression. Upregulation of 91H expression in tumor tissues associates with OS of CRC patients 20, and HOTAIR, with an antioncogenic function, inhibits the growth and migration of cancer 22. These lncRNAs are regarded as a strong prognostic indicator to predict clinical outcomes of patients 20, 22.

Sprouty4‐Intron 1 (SPRY4‐IT1, GenBank accession ID AK024556) is also a lncRNA > 680 nucleotides in length, which is first identified in adipose tissue and transcribed from the second intron of SPRY4 gene. Previous studies have shown that SPRY4‐IT1 affect melanoma cell growth, migration, and invasiveness 23, 24, 25. However, prognostic value of lncRNA SPRY4‐IT1 in melanoma patients is still unclear. Here, we evaluated the clinical significance of SPRY4‐IT1 in the plasma for patients with melanoma and healthy controls, and constructed a predictive model to predict clinical outcomes of patients.

## Materials and methods

### Patients and blood samples

Seventy blood samples were obtained from patients with malignant melanoma prior to the treatment at The People's Hospital of Chizhou, The First Affiliated Hospital, Anhui Medical University and other hospitals in Anhui Province, between 2007 and 2010. Blood‐detected SPRY4‐IT1 expression levels in 70 patients with malignant melanoma were compared with 79 healthy controls, recruited from healthy volunteers without evidence of tumor. All blood samples were handled within 30 min. All cases were confirmed primary malignant melanoma by histology. Some clinical characteristics of enrolled patients were collected in Table 1. After primary diagnosis, each individual was followed up termly until April 2015 (every 3 months for the first 2 years and subsequently every 6 months up to fifth year). OS was counted from first diagnosis to death. The date of the last follow‐up was used for drop‐out patients.

**Table 1:** Comparison between SPRY4‐IT1 expression and clinical characteristics

Variables	No. (*n* = 70) *N* (%)	SPRY‐IT1 expression^b^		*P* *
		Low expression (*n* = 38) *N* (%)	High expression (*n* = 32) *N* (%)	
Sex				
Male	45 (64.3)	26 (68.4)	19 (59.4)	0.431
Female	25 (35.7)	12 (31.6)	13 (40.6)	
Age (years)				
< 60	42 (60.0)	24 (63.2)	18 (56.3)	0.557
≥ 60	28 (40.0)	14 (36.8)	14 (43.7)	
Tumor site				
Extremities	23 (32.9)	18 (47.4)	5 (15.6)	0.019
Trunk	37 (52.9)	16 (42.1)	21 (65.6)	
Head and neck	10 (14.3)	4 (10.5)	6 (18.8)	
Histologic type				
Superficial spreading	39 (55.7)	21 (55.3)	18 (56.3)	0.934
Nodular	31 (44.3)	17 (44.7)	14 (43.7)	
Tumor stage^a^				
I–II	32 (45.7)	28 (73.7)	4 (12.5)	< 0.001
III	25 (35.7)	7 (18.4)	18 (56.3)	
IV	13 (18.9)	3 (7.9)	10 (31.3)	

*Two‐side chi‐square test.

^a^Tumor stage system according to AJCC classification.

^b^Low and high SPRY4‐IT1 groups were split by the cutoff value 2.64.

Patients enrolled in this study provided written informed consent. This experimental protocol was approved by the Medical Ethics Committee of The People's Hospital of Chizhou (Chizhou, China).

### Isolation of blood samples

Blood samples were drawn from the peripheral venous blood of each individuals and kept at 4 °C. Subsequently, 2 mL of blood sample were centrifuged at 160 g for 10 min and the supernatant fluids were further centrifuged at 4 °C, 12 000 ***g***, for 15 min in centrifuge tubes. Isolated supernatant fluids were immediately added with 1 mL of Trizol LS Regent (Invitrogen, Carlsbad, CA, USA) and stored at −80 °C until RNA extraction.

### RNA extraction and cDNA synthesis

Total RNA from the plasma of malignant melanoma, healthy controls was isolated by Trizol LS regent according to the manufacturer protocol and stored at −80 °C. RNA concentration and purity were assessed on a Nanodrop spectrophotometer (Thermo Scientific, Waltham, MA, USA). All samples were used to perform the next step when their OD_260/280_ varied from 1.8 to 2.0. cDNA synthesis used PrimeScript RT reagent Kit with gDNA Eraser (Takara, China) and was conducted for SPRY4‐IT1 levels analysis by quantitative real‐time PCR (qPCR). The cDNA was kept at −20 °C.

### Quantitative real‐time PCR

Quantitative PCR was used to determine the expression of SPRY4‐IT1 by ABI 7500 System (Applied Biosystems, Foster City, CA, USA) and SYBR Premix Ex Tag^™^ II (Takara, China) following the manufacturer recommendation. The PCR reactions were conducted in a volume of 30 μL, including 30 ng of cDNA for each sample. The PCR cycling program was set as follows: primary hold at 95 °C for 10 min, followed by 40 amplification cycles of melting at 95 °C for 15 s, annealing and extension at 60 °C.

For the normalization of blood donor data, β‐actin served as the internal control. The sequence of SPRY4‐IT1 primer was as follows: forward: 5′‐ATCCGAAGCGCAGACACAATTCA‐3′; reverse: 5′‐CCTCGATGTAGTCTATGTC ATAGGA‐3′. SPRY4‐IT1 expression levels were normalized to β‐actin to achieve the relative cycle (ΔC_T_). The relative expression was calculated by the comparative C_T_ (ΔΔC_T_) method, and then calculated relative expression folds (2^−ΔΔCT^).

### Statistical analysis

We determined the optimal cutoff value of SPRY4‐IT1 in cancerous/noncancerous by the receiver operating characteristic (ROC) curve analysis. Chi‐square test or Fisher's exact test was used to evaluate categorical data, and independent *t*‐test or Mann–Whitney *U* test analyzed continuous data. Continuous data were presented as mean ± SD. Survival curves were depicted by the Kaplan–Meier method and the significance was assessed by the Log‐rank test. Predictors for OS were determined by Univariate analysis and multivariate analysis using Cox's proportional hazards model. Prognostic nomogram was constructed by r 3.0.3 software (Institute for Statistics and Mathematics, Austria), and Harrell's concordance index (c‐index) was used to evaluate the predictive accuracy. Data analyses were performed by spss 18.0 Software (IBM, San Jose, CA, USA). *P* < 0.05 was considered statistically significant.

## Results

### Characteristics of study population

In total, 70 patients with histologically confirmed malignant melanoma were involved in this study between January 2007 and June 2010. The median follow‐up period was 52 months (range: 3–60 months). Clinical characteristics of patients who provided blood samples (melanoma patients) are depicted in Table 1. Median age of melanoma patients was 60 years (range 35–78), including 45 (64.3%) males and 25 (35.7%) females. Seventy‐nine healthy controls were of similar age and sex distribution as patients with malignant melanoma. On the basis of TNM‐stging criteria, the number of stage I–II, III, and IV was 32 (45.7%), 25 (35.7%), and 13 (18.9%), respectively. Among them, 36 melanoma patients were died from cancer‐related disease. The median of OS was 39 months in this study.

### SPRY4‐IT1 relative expression in blood of melanoma patients versus healthy controls

SPRY4‐IT1 relative expression was determined by qPCR for 70 blood donors and 79 healthy controls. Significantly higher SPRY4‐IT1 relative expression was observed in melanoma patients (mean ΔC_T_: −5.12 ± 0.62) as compared to controls (mean ΔC_T_: −4.01 ± 0.34, *P* < 0.001; Fig. 1). Subsequently, ROC curve, using OS as the end‐point for SPRY4‐IT1 relative expression, was illustrated in Fig. 2. ROC analysis exhibited area under curve (AUC) was 0.813 (*P* < 0.001) at 72.2% sensitivity and 82.4% specificity of tumor prediction, respectively. The optimal cutoff level based on OS was determined to be 2.64‐fold for SPRY4‐IT1 relative expression in cancerous/noncancerous. Patients with melanoma were divided into two groups based on the optimal cutoff level, with the high group > 2.64 (*n* = 32) and the low group < 2.64 (*n* = 38).

**Figure 1:** Comparison of lncRNA SPRY4‐IT1 in plasma of melanoma patients (*N* = 70) and healthy controls (*N* = 79). SPRY4‐IT1 expression was markedly increased in melanoma patients compared to that in healthy controls. *P < 0.01.

**Figure 2:** Cutoff value of SPRY4‐IT1 expression defined by ROC curve for overall survival.

To investigate the association of SPRY4‐IT1 expression with clinical variables, comparison between the high and low groups for SPRY4‐IT1 expression was conducted (Table 1). SPRY4‐IT1 expression was significantly associated with tumor site and TNM stage (*P*_all_ < 0.05). However, SPRY4‐IT1 expression levels were hardly related with patients' sex, age, and histologic type.

### Association of SPRY4‐IT1 relative expression with patients' prognosis

To study the association of SPRY4‐IT1 relative expression with melanoma patients' prognosis, Kaplan–Meier survival analysis and log‐rank tests were carried out. Figure 3 showed that patients with high SPRY4‐IT1 expression had a significantly poorer prognosis than those with low SPRY4‐IT1 expression (median survival time: 38 months vs. 51 months, respectively, *P* < 0.001).

**Figure 3:** Kaplan–Meier overall survival of 70 patients with melanoma stratified for high and low SPRY4‐IT1 expression. Melanoma patients with high SPRY4‐IT1 expression had shorter survival than those with low SPRY4‐IT1 expression.

Clinical variables for prediction of clinical prognosis were further investigated by univariate analysis with the Cox regression model. The significant variables in univariate analysis combined with sex and age were then investigated for the impact on OS by multivariate analysis. Our results revealed that elevated SPRY4‐IT1 expression, tumor in head and neck, and advanced TNM stage were obviously associated with the worse OS. Furthermore, SPRY4‐IT1 relative expression was considered to be an independent prognostic factor for OS in patients with melanoma (Table 2).

**Table 2:** Cox proportional hazard analysis: impact of SPRY4‐IT1 and clinical variables on overall survival in melanoma patients

Variables	Category	Overall survival					
		Univariate analysis			Multivariate analysis		
		HR	95% CI	*P*	HR	95% CI	*P*
Sex	Male	1					
	Female	1.026	0.520–2.027	0.940			
Age (years)	< 60	1					
	≥ 60	1.078	0.556–2.092	0.823			
Tumor site	Extremities	1			1		
	Trunk	1.794	0.793–4.060	0.161	1.025	0.433–2.424	0.956
	Head and neck	2.949	1.064–8.170	0.038	1.973	0.682–5.705	0.210
Histologic type	Superficial spreading	1					
	Nodular	1.066	0.554–2.053	0.849			
Tumor stage^a^	I‐II	1			1		
	III	3.842	1.638–9.011	0.002	1.789	0.608–5.269	0.291
	IV	5.21	2.120–12.806	< 0.001	2.507	1.021–7.305	0.047
SPRY‐IT1 expression^b^	Low	1			1		
	High	4.801	2.292–10.060	< 0.001	2.931	1.103–7.790	0.031

a Tumor stage system according to AJCC classification.

b Low and high SPRY4‐IT1 groups were split by the cutoff value 2.64.

To predict clinical outcomes of patients with malignant melanoma after primary diagnosis, predictive model was established combining all significant clinical characteristics in multivariate analysis (Fig. 4A). The nomogram would predict the probability of 5‐year survival for melanoma patients after first diagnosis (c‐index: 0.72). In addition, we also performed internal calibration that shows the predictions from nomogram compared to actual outcomes for 70 patients with melanoma. The calibration curve shows a good predictive match with the actual outcomes (Fig. 4B).

**Figure 4:** Nomogram for survival of patients with melanoma prior to treatment (A); calibration curve for 5‐year survival (B). The solid line refers to performance of the actual nomogram, and the dashed line shows an ideal nomogram.

## Discussion

Malignant melanoma is a most aggressive malignancy among all skin cancers 1. Most patients are diagnosed at an advanced stage, and many treatments for melanoma are therefore less effective. It is necessary to find a useful marker to diagnose early and improve the prognosis of malignant melanoma. Hence, a better understanding of this cancer contributes to find a surrogate marker to predict the progression and prognosis of melanoma, which may lead to improvement in the diagnosis and treatment of malignant melanoma.

In this study, we evaluated the expression levels of SPRY4‐IT1 in the plasma of patients with melanoma and healthy controls by qRT‐PCR for the first time, and explored clinical significance of SPRY4‐IT1 in melanoma patients. The results showed that lncRNA SPRY4‐IT1 was upregulated in melanoma patients compared to healthy controls. We also found that SPRY4‐IT1 expression was associated with tumor site and tumor stage of patients with melanoma. Furthermore, relative expression levels of SPRY4‐IT1 were not linked with patients' sex, age, and histologic type. Upregulation of SPRY4‐IT1 expression is negatively correlated with overall survival rates and was an independent factor in patients with melanoma. Our established model could predict clinical outcomes of patients with melanoma. These results reveal that SPRY4‐IT1 may play a critical role in the progression and prognosis of malignant melanoma, and it may be regarded as a surrogate prognostic marker for melanoma.

LncRNAs, > 200 nt in length, are generally defined as transcribed RNA molecules, lack of potential protein‐coding capacity 26. Emerging evidence has shown that lncRNAs may be emerged as key regulators of important biologic cellular processes and multiple diseases 27, 28. Increasing lncRNAs have been identified to play an essential role in the carcinogenesis and progression 29, 30. At present, some hot lncRNAs have been deeply explored, including HOX antisense intergenic RNA (HOTAIR), metastasis‐associated lung adenocarcinoma transcript 1 (MALAT1), and maternally expressed 3 (MEG3).

SPRY4‐IT1 is first identified to be differentially expressed in melanoma cells, and it is transcribed from an intron of the SPRY4 gene containing several long hairpins in its secondary structure. SPRY4‐IT1 knockdown results in the inhibition of biologic behaviors in melanoma cells 23. Subsequently, Xie and colleagues reported that lncRNA SPRY4‐IT1 is overexpressed in esophageal squamous cell carcinoma and associates with poor prognosis 31. Moreover, lncRNA SPRY4‐IT1 has been reported to play an important role in various types of cancers, including prostate cancer 32, glioma 33, and gastric cancer 34. Previous reports indicated that SPRY4‐IT1 regulates the growth and metastasis of many cancers. In our study, we found that SPRY4‐IT1 expression levels is strongly associated with tumor stage and clinical prognosis. Nomogram has been identified to be more precise than the traditional AJCC staging system for predicting clinical outcomes in malignancies, especially prostate cancer 35.

Prognostic model can help physicians to identify high‐risk patients to improve the treatment and prognosis of patients. Nomogram has been developed to predict clinical outcomes in patients with various types of malignancies 36, 37. Tumor stage can be used to evaluate patients' outcomes according to risk for their disease progression and death. We are also attempting to develop a predictive model to predict the probability of 5‐year overall survival for patients with melanoma according to lncRNA and the significant factors in multivariate analysis. Our constructive model was performed well in predicting the clinical prognosis of patients with melanoma based on the c‐index and calibration curve. The purpose of this model is to calculate some of the heterogeneity within the tumor stages and provide a precise predictor for survival.

Although this study provides a new approach into the evaluation of clinical outcomes for melanoma patients, some limitations should be acknowledged. First, the relative expression of SPRY4‐IT1 in tissue samples is not estimated because of unavailable tissue samples. Second, the results derived from 70 patients with melanoma and 79 healthy controls are limited and need to be identified by other studies with large samples.

Third, we could not exclude some heterogeneity of treatments to lead to differentiation of clinical prognosis.

In conclusion, for the first time, we have demonstrated that lncRNA SPRY4‐IT1 is overexpressed in the plasma for patients with malignant melanoma compared to that in healthy controls. Dysregulation of SPRY4‐IT1 is closely associated with tumor site, tumor stage, and clinical outcomes. These findings support that SPRY4‐IT1 may be a potential prognostic marker for functioning as surveillance and prediction of prognosis in malignant melanoma.

## Author contributions

TL and ZGL conceived and designed the experiments. TL, SKS, JGX, YX, HQZ, and HJL performed the experiments. TL and SKS analyzed the data. SKS, JGX, HQZ, and HJL contributed reagents/materials/analysis tools. TL and ZGL wrote the manuscript.
